The article "Novel C‐terminal heat shock protein 90 inhibitors target breast cancer stem cells and block migration, self‐renewal, and epithelial–mesenchymal transition" was retracted in 2026. Reasons: duplicated images; unreliable results or conclusions.

# Novel C‐terminal heat shock protein 90 inhibitors target breast cancer stem cells and block migration, self‐renewal, and epithelial–mesenchymal transition

**DOI:** 10.1002/1878-0261.12686

**Published:** 2020-05-15

**Authors:** Chitra Subramanian, Patrick T. Grogan, Ton Wang, Joseph Bazzill, Ang Zuo, Peter T. White, Avinaash Kalidindi, Dawn Kuszynski, Grace Wang, Brian S. J. Blagg, Mark S. Cohen

**Affiliations:** ^1^ Department of Surgery University of Michigan Ann Arbor MI USA; ^2^ Division of Hematology Medical Oncology, and Palliative Care University of Wisconsin Madison WI USA; ^3^ Department of Pharmaceutical Sciences University of Michigan Ann Arbor MI USA; ^4^ Department of Chemistry and Biochemistry University of Notre Dame IN USA; ^5^ Department of Pathology University of Michigan Ann Arbor MI USA; ^6^ Department of Pharmacology University of Michigan Ann Arbor MI USA; ^7^ Department of Biomedical Engineering University of Michigan Ann Arbor MI USA

**Keywords:** heat shock protein 90 inhibitor, triple‐negative breast cancer, tumor‐initiating cells

## Abstract

In patients with triple‐negative breast cancer (TNBC), evidence suggests that tumor‐initiating cells (TIC) have stem cell‐like properties, leading to invasion and metastasis. HSP90 plays a critical role in the conformational maintenance of many client proteins in TIC development. Therefore, we hypothesize that the novel C‐terminal HSP90 inhibitors KU711 and KU758 can target TIC and represent a promising strategy for overcoming metastasis. Human breast cancer cells (MDA‐MB‐468LN, MDA‐MB‐231) treated with the HSP90 inhibitors KU711, KU758, and 17‐AAG showed a 50–80% decrease in TIC markers CD44 and aldehyde dehydrogenase (*P* < 0.01) as assessed by flow cytometry. A decrease in sphere formation, which was used to assess self‐renewal, was observed after the treatment of TNBC cells starting at 2.5 µm KU711 and 0.31 µm KU758. KU compounds also blocked the invasion and migration of TNBC cells in a dose‐dependent manner. The knockdown of HSP90 clients was observed without any change in prosurvival HSP70 levels. *In vivo,* in a murine orthotopic breast cancer model, treatment with KU758 and KU711 yielded an approximately twofold and a fourfold reduction in tumor volumes versus control, respectively, without demonstrated toxicity. In conclusion, C‐terminal HSP90 inhibitors are potent novel therapeutics against TNBC *in vitro* and *in vivo* as they target TICs and block invasion, EMT transition, and self‐renewal.

## Graphical abstract

C‐terminal HSP90 inhibitors KU711 and KU758 reduce tumor growth of triple‐negative breast cancer xenografts by targeting Akt/mTOR and MAPK/ERK pathways, cancer stem cells, migration, and EMT transition.

**Abbreviations**
17‐AAG: 17‐*N*‐allylamino‐17‐demethoxygeldanamycin
ALDH: aldehyde dehydrogenase
HER2/neu: human epidermal growth factor
HSP90: heat shock protein 90
OS: overall survival
TIC: tumor‐initiating cells
TNBC: triple‐negative breast cancer

## 1 Introduction

In the United States, breast cancer was responsible for ~ 40 000 deaths in 2018 and is the main cause of fatality among women second only to lung cancer (Jemal *et al.*, 2010). Although advances in early detection and treatment with adjuvant therapies have improved the survival rate of different types of breast cancer, treatment of triple‐negative breast cancer (TNBC) remains challenging, and this subset of patients has poor clinical prognoses compared to other breast cancer subtypes (Nagamatsu *et al.*, 2014). Approximately 10–20% of breast cancer patients who are diagnosed with TNBC lack expression of estrogen receptor, progesterone receptor, and human epidermal growth factor (HER2/neu) (Carey *et al.*, 2006). With no targeted therapies currently available for treating TNBCs, systemic chemotherapy remains the mainstay of treatment for both early‐stage and advanced patients. Although TNBC patients respond well to chemotherapy initially, many are at high risk of metastatic recurrence and have poor outcomes (Liedtke *et al.*, 2008). Hence, the development of novel therapeutic strategies for improving the overall survival (OS) of TNBC patients is urgently needed.

Emerging evidence suggests that a small population of cells that have stem cell‐like properties escape treatment, which leads to invasion and metastasis, treatment resistance, and recurrence in breast cancer (Charafe‐Jauffret *et al.*, 2009; Morrison *et al.*, 2011). These populations of cells are known as cancer stem cells or tumor‐initiating cells (TICs) and are defined by the expression of markers such as CD44^+^/CD24^−^, aldehyde dehydrogenase (ALDH), and others (Ginestier *et al.*, 2007; Luo *et al.*, 2015). Signaling pathways like hedgehog, notch, WNT, interleukin 6/STAT3, IL8/CXCR1/2, TGFβ, and integrin are known to regulate TICs and lead to therapy resistance (Wei and Lewis, 2015). Heat shock proteins (HSP90 and HSP70) play a critical role in the folding and conformational maintenance of a diverse set of client proteins involved in TIC developmental pathways including kinases, transcription factors, and other proteins (Chiosis and Neckers, 2006). Therefore, HSP90 inhibitors that downregulate these essential pathways for breast TIC function represent a promising strategy for overcoming therapy failure, recurrence, and metastasis.

Currently, blocking the function of heat shock protein 90 (HSP90) using small molecules has shown encouraging results in phase I/II clinical trials for several cancers including breast cancer (Solarova *et al.*, 2015). The ubiquitously expressed HSP90 functions as a master switch and controls late‐stage maturation, activation, and stability of numerous cellular protein clients that are implicated in the pathogenesis of breast cancer (Neckers and Workman, 2012). The geldanamycin derivative 17‐*N*‐allylamino‐17‐demethoxygeldanamycin (17‐AAG) binds to the N‐terminal ATP binding site of HSP90 and initially demonstrated clinical benefit in several cancers. However, 17‐AAG did not pass phase II trials owing to poor solubility, low oral bioavailability, metabolic issues, and hepatic toxicity (Egorin *et al.*, 2001; Guo *et al.*, 2005). To overcome the limitations of 17‐AAG, several small‐molecule N‐terminal HSP90 inhibitors were developed and are in clinical trials for cancer. All of these compounds have struggled with challenges related to the induction of the prosurvival heat shock response, liver toxicity, and drug resistance, dampening the development of HSP90 inhibitors as potential anticancer therapeutics.

To overcome the drawbacks of the N‐terminal HSP90 inhibitors, we have developed several novel novobiocin analogues as C‐terminal HSP90 inhibitors and have examined their efficacy in targeting multiple cancer models including breast cancer (Zhao *et al.*, 2014). Contrary to the N‐terminal inhibitors that are in clinical trials, these C‐terminal inhibitors do not induce the prosurvival heat shock response. In the current study, we evaluate the mechanism through which two novel analogues of novobiocin, namely KU711 and KU758, target TNBC both *in vitro* and *in vivo.* Our results indicate that the novel KU compounds KU711 and KU758 are highly effective in targeting cancer stem cells, preventing sphere formation, migration, invasion, and EMT transition by targeting HSP90 clients, and cause tumor regression *in vivo*.

## 2 Materials and methods

### 2.1 Cell lines and reagents

Validated human TNBC cell lines MDA‐MB‐231 (Claudin‐low) and MDA‐MB‐468LN (basal) (Vantyghem *et al.*, 2005) were grown in Dulbecco’s modified Eagle’s medium (Life Technologies, Carlsbad, CA, USA) supplemented with 10% FBS (Sigma‐Aldrich, St. Louis, MO, USA) and 1% penicillin/streptomycin (Life Technologies). Novel C‐terminal HSP90 inhibitors KU711 and KU758 (Fig. 1) were provided by Dr B. S. J. Blagg (University of Notre Dame), and the N‐terminal HSP90 inhibitor 17‐AAG was obtained from Sigma‐Aldrich.

**Fig. 1:** Schematic representation of the structure of KU711 and KU758.

### 2.2 Mammosphere formation assay

Approximately 250 TNBC cells (either MDA‐MB‐231 or MDA‐MB‐468LN) per well were plated in an ultralow attachment 96‐well tissue culture plates (Corning, Tewksbury, MA, USA). The cells were then treated with multiple concentrations of KU711 (2.5–40 µm) and KU758 (0.3125–5.0 µm) in MammoCult (human) complete medium (STEMCELL Technologies, Vancouver, Canada). After 5 days, spheres greater than 50 cells were counted using light microscopy.

### 2.3 Boyden chamber migration and invasion assay

Approximately 1 × 10^5^ TNBC cells (MDA‐MB‐231 or MDA‐MB‐468LN) suspended in serum‐free medium containing the drugs (20–40 μm KU711, 2.5–5 μm KU758, and 2.0 μm 17‐AAG) were seeded into the upper wells of an 8‐micron polycarbonate transwell chamber (Corning). The Boyden chambers were placed in a 24‐well plate containing 10% FBS as a chemoattractant. The standard Boyden chambers were used for the evaluation of migration, whereas for examining the invasion, the wells were coated with 100 µL of 300 µg·mL^−1^ of reduced growth factor Matrigel (Corning). The chambers were incubated for 24 h, and the cells that had invaded to the bottom of the chamber were fixed (2% paraformaldehyde), stained (1% crystal violet in 20% methanol) for 20 min., washed, and counted after the removal of noninvaded cells using a cotton swab using an inverted microscope. Each experiment was done in triplicate.

### 2.4 Flow cytometry

MDA‐MB‐231 and MDA‐MB‐468LN cells were treated with varying concentrations of KU711 (20–40 μm), KU758 (1.0–2.5 μm), and 17‐AAG (2.0 μm) for 24 h. Cells were collected and then stained first for ALDEFLUOR as per the manufacturer’s instruction (STEMCELL Technologies) followed by CD44−APC (BD Biosciences, San Jose, CA, USA), and then evaluated for ALDH activity and CD44 levels by flow cytometry using CyAn ADP analyzer (Beckman Coulter, Brea, CA, USA). Diethylaminobenzaldehyde was used as a negative control for the ALDEFLUOR assay.

### 2.5 Western blot analysis

MDA‐MB‐468LN grown to 60–80% confluence was treated with varying concentrations of HSP90 inhibitors (KU711 and KU758) and 17‐AAG for 24 h. Proteins extracted from the cells post‐treatment were quantified using BCA protein assay (Thermo Fisher Scientific, Waltham, MA, USA). To isolate protein from tumor samples, the tumors were sonicated and lysed and the proteins were isolated as previously described (Samadi *et al.*, 2010). Equal amount of proteins separated on a SDS/PAGE was then transferred on to a nitrocellulose membrane and western blotted for HSP90 client proteins as previously described (Subramanian *et al.*, 2014). As a loading control, actin or GAPDH was used and all experiments were repeated for accuracy. Densitometric analyses of protein expression were performed using imagej software from (NIH, Bethesda, MD, USA).

### 2.6 *In vivo* breast tumor xenograft

Approximately 6‐ to 8‐week‐old female athymic nude nu/nu mice (Harlan Laboratories, Indianapolis, IN, USA) received a mammary fat pad injection of 3 × 10^6^ MDA‐MB‐468LN cells in 100 μL of sterile 1× PBS. The mice were randomly divided into treatment groups of 10 mice per group (Control, KU711, KU758, and 17‐AAG) when the tumor size was ~ 50 mm^3^. The treatment group mice received intraperitoneal injection of the drugs [KU711 (5 mg·kg^−1^·d^−1^), KU758 (5 mg·kg^−1^/thrice weekly), 17‐AAG (50 mg·kg^−1^·d^−1^), and control dimethyl sulfoxide (DMSO) groups] for 21 days. KU758 was used thrice weekly due to toxicity associated with daily administration of the drug. The weight of the mice was observed thrice weekly to evaluate the general toxicity of the treatment. Simultaneously, the tumor volume was measured using a digital caliper. The formula used for the tumor volume calculation was as follows: length × (width)^2^ × π/6. The animals were followed for an additional 4 weeks post‐treatment, and tumor volume and weight were measured. At the end of the treatment, two mice from each group were randomly euthanized to evaluate protein changes and for histology (Samadi *et al.*, 2010). Animal survival was monitored with animals removed from the study at morbidity or death, and a Kaplan–Meier survival curve was plotted using graphpad prism software (San Diego, CA, USA). Morbidity was characterized by a body condition score of < 2 or a tumor burden impairing animal mobility or functioning. To evaluate whether changes in CD44 levels seen *in vitro* can be recapitulated *in vivo*, we examined tumor samples explanted from two mice after treatment with KU711, KU758, or 17‐AAG. CD44 levels were evaluated by western blot, and immunohistochemical analysis of the tumor samples was performed for the proliferation marker Ki‐67. All experiments involving mice were carried out according to the University Committee on Use and Care of Animals (UCUCA) protocol at the University of Michigan.

### 2.7 Statistical analysis

To estimate the significance between different treatments, Student’s two‐tailed, unpaired *t*‐test was used in mammosphere assays, flow cytometry, and Boyden chamber assays. Data were graphed as mean values with standard deviation as error bars. For accuracy, the experiments were repeated thrice. Biostatistical data points were determined throughout the *in vivo* study, and tumor volumes and animal masses were calculated as mean ± SE. Treatment differences with respect to tumor size were assessed using two‐way ANOVA with a *post hoc* nonparametric test in prism software. Excel software was used to plot the tumor volume progression/regression. A *P*‐value of less than 0.05 was used as statistically significant.

## 3 Results

### 3.1 Treatment of TNBC cells with C‐terminal HSP90 inhibitor KU711 or KU758 reduces the number of mammospheres, migration, and invasion of TNBC cells

Breast cancer TICs are implicated in the recurrence and metastasis of breast cancer. Therefore, to evaluate the efficacy of the novel C‐terminal HSP90 inhibitors KU711 and KU758 in targeting breast cancer TICs, two TNBC cell lines MDA‐MB‐468LN and MDA‐MB‐231 were treated with varying concentrations of KU711 and KU758 starting from 2.5 µm KU711 and 0.3125 µm KU758. As seen in Fig. 2A, when TNBC cells were treated with HSP90 inhibitors, we observed a dose‐dependent decrease in sphere formation. In MDA‐MB‐468LN cells, there is a significant decrease in sphere formation with even the lowest dose of KU711 and KU758 treatment (*P* < 0.04), with > 90% self‐renewal inhibition at doses of 40 µm KU711 and 2.5 µm KU758. In MDA‐MB‐231 cells, there is a significant decrease in sphere formation with the lowest dose of KU711, and from 1.25 µm KU758 (*P* < 0.03) with > 90% self‐renewal inhibition at doses of 40 µm KU711 and 5.0 µm KU758. By comparison, treatment with 2.0 µm of the N‐terminal HSP90 inhibitor 17‐AAG results in a lesser, but still significant decrease in sphere formation between 15% and 76% compared to control in TNBC cells (*P* < 0.01). Sphere formation in MDA‐MB‐468LN cells after treatment with HSP90 inhibition is shown in Fig. 2B. Next, we examined whether treatment of TNBC cells with the C‐terminal HSP90 inhibitors is able to inhibit cellular migration and invasion. MDA‐MB‐468LN and MDA‐MB‐231 cell lines were treated with increasing concentrations of KU711 (20–40 µm), KU758 (2.5–5.0 µm), and 2.0 µm 17‐AAG, and migration and invasion of the cells through Boyden chamber and Matrigel were assessed. As shown in Fig. 2C, treatment of TNBC cell lines with KU711 and KU758 results in a dose‐dependent decrease in migration compared to control (between 40% and 100% for KU711, 94% and 100% for KU758, and 67% and 70% for 17‐AAG; *P* < 0.01). Similarly, there is a dose‐dependent decrease in invasion compared to control (between 71% and 99% for KU711, 85% and 100% for KU758, and 81% and 100% for 17‐AAG; *P* < 0.01). Invasion and migration of MDA‐MB‐468LN cells after treatment with HSP90 inhibition are shown in Fig. 2D.

**Fig. 2:** (A, C) TBNC cells MDA‐MB‐231 and MDA‐MB‐468LN were treated with KU711, KU758, and 17‐AAG for 24 h. Percent sphere formation (A), migration, and invasion (C) compared to control are shown. (B, D) Treatment of MDA‐MB‐468LN cells with KU711, KU758, and 17‐AAG for 24 h decreases mammosphere formation (B) Scale bars: 100 µm); and migration and invasion (D, Scale bars: 200 µm) in a dose‐dependent manner. Each experiment was repeated thrice, and the values were represented as mean ± SD. The statistical significance was calculated by Student’s two‐tailed, unpaired *t*‐test, and *P* < 0.05 was set as significant value. ** represents *P* ≤ 0.01.

### 3.2 The C‐terminal HSP90 inhibitors KU711 and KU758 reduce the expression of TIC markers CD44 and ALDH

CD44 and ALDH are known as potential markers for the presence of breast cancer stem cells. Hence, we next examined whether KU711 and KU758 treatment of TNBC cells would result in changes in the expression of CD44 and ALDH by flow cytometry. As shown in Fig. 3A,B, treatment of MDA‐MB‐468 LN cells with 20–40 µm KU711 and 1–2.5 µm KU758 resulted in a 25–85% and 81–95% decrease in the TIC marker ALDH (*P* < 0.03), respectively. This result was further confirmed by measuring the mean fluorescent intensity for ALDH, which showed a 29–95%, 21–97%, and 3% decrease after treatment with 20–40 µm KU711, 1–2.5 µm KU758, and 2.0 µm 17‐AAG, respectively (*P* < 0.05). Similarly, treatment with 20–40 µm KU711 and 1–2.5 µm KU758 resulted in a 22–73% and 31–49% decrease in the TIC marker CD44 (*P* < 0.01), respectively. By comparison, treatment with 2.0 µm 17‐AAG resulted in a 51% and 4% decrease in ALDH and CD44, respectively (*P* < 0.01 for ALDH).

**Fig. 3:** (A, B) Treatment of MDA‐MB‐468 LN cells with varying concentrations of the HSP90 inhibitors KU711, KU758, and 17‐AAG for 24 h decreases the levels of TIC markers CD44 and ALDH. Each experiment was repeated thrice, and the values were represented as mean ± SD. The statistical significance was calculated by Student’s two‐tailed, unpaired *t*‐test, and *P* < 0.05 was set as significant value. ** represents *P* ≤ 0.01.

### 3.3 KU711 and KU758 reduce the levels of cancer stem cell markers and EMT

MDA‐MB‐468 LN cells were treated with increasing concentrations of KU711 (10–40 µm), KU758 (1.0–5.0 µm), and 17‐AAG (2.0 µm) for 24 h. The cells were lysed and immunoblotted for BMI‐1, EZH2, and vimentin. As shown in Fig. 4, EZH2 levels decreased with increasing concentrations of C‐terminal inhibitor treatment for both KU711 and KU758 to a greater extent than treatment with the N‐terminal inhibitor 17‐AAG. EZH2 is important in histone methylation and epigenetic modification of its downstream targets. Importantly, EZH2 is upregulated in many cancers, including breast cancer, and is important in tumor cell and cancer stem cell proliferation and subsequent metastasis. Additionally, there is a dose‐dependent decrease in the levels of BMI‐1 with increasing concentrations of treatment with KU711 and KU758, which is more striking than with treatment with 17‐AAG. BMI‐1 is an oncogene that is part of the polycomb group, and its role in normal stem and tumor stem cell proliferation has been previously described. Notably, depletion of BMI‐1 from progenitor cells results in apoptosis and proliferative arrest. Finally, treatment of breast cancer cells with KU711 and KU758 leads to a dose‐dependent decrease in vimentin, a well‐known marker of epithelial‐to‐mesenchymal transition. Taken as a whole, these findings suggest that the C‐terminal specific compounds KU758 and KU711 are able to suppress cancer stem cell proliferation and epithelial‐to‐mesenchymal transition, two important processes that are thought to contribute to the metastatic spread of disease. Importantly, the suppressive effect of our novel C‐terminal inhibitors is greater than that from the classic N‐terminal inhibitor 17‐AAG. Actin levels are shown as a loading control.

**Fig. 4:** MDA‐MB‐468LN cells were treated with the HSP90 inhibitors KU711, KU758, and 17‐AAG for 24 h. The cells were lysed and immunoblotted for BMI‐1, EZH2, and vimentin. Both C‐terminal inhibitors reduce the levels of cancer stem cell markers and EMT. Actin is shown as a loading control.

### 3.4 KU711 and KU758 alter the levels of proteins involved in multiple oncogenic pathways without induction of the heat shock response

MDA‐MB‐468 LN cells were treated with varying concentrations of C‐terminal HSP90 inhibitors KU711 (0.01–25 µm) and KU758 (0.01–1.0 µm) as well as the N‐terminal HSP90 inhibitor 17‐AAG (1.0 µm) for 24 h. The cells were collected, lysed, and immunoblotted for HSP90 client proteins to evaluate modulation of oncogenic pathways implicated in the development of breast TICs. As shown in Fig. 5A, there is a dose‐dependent decrease in mTOR, p‐mTOR, Akt, and p‐Akt with treatment with both KU711 and KU758. Densitometric analyses of protein expression showed a dose‐dependent decrease in p‐Akt after treatment with KU711, KU758, and 17‐AAG (Fig. 5B). Additionally, there is a dose‐dependent decrease in Cdk4 and Cdk6 with treatment with KU711 and KU758. The Cdk4/6 pathway is important in the regulation of the cell cycle transition from G1 to S phases and has been a key target for novel breast cancer therapies due to its frequent dysregulation in breast cancer cells. Conversely, treatment with KU758 and KU711 appears to increase the expression of p‐ERK1/2; there is no difference in the expression of ERK2. ERK activation has been shown to play vital roles in both cell survival and apoptotic pathways (Mebratu and Tesfaigzi, 2009). Induction of apoptosis with increased ERK phosphorylation suggests that the HSP90 inhibitors KU711 and KU758 are involved in the cell death mechanism of ERK activation. This is further confirmed by the densitometric analyses, as shown in Fig. 5B. Treatment with KU758 increases Raf‐1 and p‐Raf‐1 at high concentrations; there is no alteration in either level with KU711 treatment. Interestingly, the levels of BRCA1 and pBRCA decrease with KU711 treatment but increase with KU758 treatment in a dose‐dependent manner. Induction of apoptosis after treatment with drugs was analyzed by cleavage of PARP and caspase 7. Importantly, with treatment of KU758 and KU711, there is no change in the levels of the heat shock response proteins HSP90, HSP32, and HSF1, and a decrease in HSP70 with higher concentrations, which was confirmed further by densitometric analysis. By comparison, there is an increase in HSP70 expression with 17‐AAG treatment. A significant concern with the traditional N‐terminal HSP90 inhibitors is the adverse activation of the prosurvival heat shock response, which serves to stabilize intracellular proteins and assist in refolding any damaged proteins. To test the loading efficiency, GAPDH was used.

**Fig. 5:** (A) MDA‐MB‐468LN cells were treated with varying concentrations of the HSP90 inhibitors KU711, KU758, and 17AAG for 24 h. The cells were collected, lysed, and immunoblotted for HSP90 client proteins to evaluate the modulation of pathways implicated in the development of breast TICs. Induction of apoptosis after treatment with drugs was analyzed by cleavage of PARP, caspase 3, and caspase 7. To test the loading efficiency, GAPDH was used. (B) Densitometric analysis was done using imagej.

### 3.5 KU711 and KU758 are more effective compared to 17‐AAG and control at suppressing breast cancer tumor growth *in vivo*

Approximately 3 million MDA‐MB‐468LN cells were injected into the flank region of nude mice. Once the tumors reached ~ 50 mm^3^, the mice were treated with KU758, KU711, 17‐AAG, or control DMSO  for 21 days. Tumor volumes were measured three times per week for 65 days. As shown in Fig. 6A, tumor volume size at the end of the study for mice treated with KU758, KU711, and 17‐AAG was 52%, 31%, and 63%, respectively, compared to that of the control mice. At the end of treatment, tissues were collected for histological analysis to evaluate the toxicity of these compounds. Statistical analysis of tumor treatment differences for tumor size using two‐way ANOVA with a *post hoc* nonparametric test showed significant decreases in tumor volume for all the treatments compared to control mice. Of the different HSP90 inhibitor treatment groups, KU711 treatment resulted in significant changes in tumor volume (*P* < 0.05) compared to either 17‐AAG or KU758 treatment. The tissues were stained with H&E, and toxicity was analyzed by a pathologist. As shown in Fig. 6B, KU758 was associated with slight toxicity to the liver (patchy centrilobular hepatic necrosis, patchy periportal eosinophilic and lymphoplasmacytic infiltrate, hepatocyte nuclear size variability) and kidneys (mild lymphocytic junctional medullary infiltrate). However, KU711, which demonstrated the best tumor response to drug treatment, was not associated with any toxic side effects to the liver or kidneys. The Kaplan–Meier survival curve (Fig. 6C) shows a better OS rate after treatment with KU711 compared to KU758 or 17‐AAG. To evaluate whether changes in CD44 levels seen *in vitro* can be recapitulated *in vivo*, we have examined the tumor samples explanted from mice after treatment with KU711, KU758, or 17‐AAG. As shown in the western blot Fig. 7A, KU 711 and KU758 treatment resulted in ~ 22–30% and 21–65% decrease in CD44 for KU758 and KU711, respectively, whereas treatment with the N‐terminal HSP90 inhibitor 17‐AAG did not result in significant changes in CD44 levels. Immunohistochemical analysis of the tumor samples for the proliferation marker Ki‐67 (Fig. 7B) showed 18%, 35%, and 61% decrease in proliferation for 17‐AAG, KU758, and KU711, respectively. Overall, the *in vivo* study indicated that KU711 is the most effective C‐terminal HSP90 inhibitor for targeting breast cancer.

**Fig. 6:** (A) Approximately 3 million MDA‐MB‐468 LN cells were injected into the flank region of nude mice, and once the tumors reached ~ 50 mm^3^, the mice were treated either daily or twice a week for 21 days with KU711, KU758, or 17‐AAG. Tumor volumes were measured twice weekly and plotted. Six mice from each group were used, and the mean ± SE values were plotted. Treatment differences with respect to tumor size were assessed using two‐way ANOVA with a *post hoc* nonparametric test with *P* < 0.05 set as statistically significant. (B) Toxicity analysis using histology. At the end of the treatment, tissues were collected for toxicity analysis. The tissues were stained with H&E, and toxicity was analyzed by a pathologist. KU711, which demonstrated the best antitumor efficacy *in vivo*, was not toxic compared to 17‐AAG and KU758. (C) Kaplan–Meier survival curve. * represents *P* ≤ 0.05 and *** represents *P* ≤ 0.001.

**Fig. 7:** (A) C‐terminal HSP90 inhibitor treatment decreased the expression of CD44. Proteins were extracted from tumor samples from two mice treated with KU711, KU758, or 17‐AAG and one control mice. The proteins were subjected to immunoblot for CD44 (1 and 2 represent mice 1 and 2 from each group). The same blot was stripped and blotted for GAPDH as a loading control. imagej analysis was used to quantify the changes in CD44 levels in terms of GAPDH. (B) Immunohistochemistry of tumor samples of mice after treatment showed a decrease in Ki‐67 levels with KU758 and KU711 treatment, whereas 17‐AAG treatment did not result in a significant change in Ki‐67 levels (Scale bars: 200 µm). Three areas from two mice from each group were evaluated, and the values were represented as mean ± SD. The statistical significance was calculated by Student’s two‐tailed, unpaired *t*‐test, and *P* < 0.05 was set as significant value.* represents *P* ≤ 0.05 and *** represents *P* ≤ 0.001.

## 4 Discussion

Despite evaluating 18 different HSP90 inhibitors in clinical trials, there are currently no FDA‐approved HSP90 inhibitors (Yuno *et al.*, 2018). All of the tested HSP90 inhibitors to date have been N‐terminal inhibitors; 17‐AAG, 17‐DMAG, AUY922, ganetespib, and IPI‐504 have been evaluated as mono‐ or combination therapy in triple‐negative and HER2+ breast cancer. HSP90 inhibitors such as 17‐AAG in combination with trastuzumab have shown the most promise in HER2+ breast cancer because HER2 is a known client protein of HSP90 (De Mattos‐Arruda and Cortes, 2012). However, there are great rationale and preliminary data to support the investigation of using HSP90 inhibitors in TNBC as well, as many HSP90 client proteins (including AKT, EGFR, ERK) are implicated in oncogenesis. This is supported in our study, as HSP90 inhibition with KU711 and KU758 has notable effects on multiple oncogenic pathways including BRCA1, the mTOR/Akt pathway, the MAPK/ERK pathway, and the Cdk4/6 pathway, ultimately resulting in caspase cleavage and apoptosis.

A major limiting factor of utilizing HSP90 inhibitors for cancer treatment is that the concentration of HSP90 N‐terminal inhibitors required to induce client protein degradation is the same as that needed to induce the heat shock response, which results in the overexpression of both HSP70 and HSP90 and a prosurvival effect in the cell. This then requires higher doses of HSP90 inhibition to maintain the anticancer/proapoptotic effect and ultimately leads to dose‐limiting toxicity (Kim *et al.*, 2009). Thus, inhibition of HSP90 at the C‐terminal dimerization domain as opposed to the N‐terminal ATPase domain is an attractive strategy, as it has been shown that C‐terminal inhibition can cause client protein degradation without inducing the prosurvival heat shock response (Davis *et al.*, 2017). This is seen in our study, in which there is no alteration in protein levels of the heat shock proteins (HSP32, HSP70, HSF1) after treatment with the C‐terminal inhibitors KU758 and KU711, but there is upregulation of HSP70 after treatment with the N‐terminal inhibitor 17‐AAG.

The main cause of mortality for patients with TNBC is recurrent and metastatic disease. There has been much interest in studying TICs, or cancer stem cells, which have the ability to self‐renew and regenerate. In our study, we demonstrate that treatment of TNBC cells with the novel C‐terminal HSP90 inhibitors KU711 and KU758 is able to specifically target TICs. With treatment, there is decreased mammosphere formation, and flow cytometry shows a decrease in the percentage of CD44−/ALDH‐positive cells. Importantly, the decrease in the population of TICs is more prominent with treatment with C‐terminal HSP90 inhibition compared to treatment with the N‐terminal inhibitor 17‐AAG. Similar to our findings *in vitro*, we observed significant knockdown of CD44 in mice treated with KU711 and KU758 but not in mice treated with the N‐terminal HSP90 inhibitor 17‐AAG. Our results with C‐terminal HSP90 inhibitors are similar to the treatment of the TNBC cells with a deguelin derivative, L80, which showed targeting of TICs via STAT3 inhibition in TNBC cells (Cho *et al.*, 2019). Further supporting the efficacy of KU711 and KU758 at targeting TICs is the demonstrated decrease in migration and invasion and protein levels of BMI‐1, EZH2, and vimentin, which are all implicated in metastasis and epithelial–mesenchymal transition.

In this pilot study, we are able to demonstrate that KU711 and KU758 are effective in slowing TBNC tumor growth in mice after treatment for 21 days, an effect that appears durable for up to 65 days after tumor inoculation. Additionally, the average tumor volume at the end of the study was smaller in mice treated with both KU711 and KU758 compared to 17‐AAG. KU711, which had the best effect on tumor volume, was not associated with any toxic side effects, and KU758 showed only minimal side effects on kidney and liver histology. In addition to dramatically smaller average tumor size (50% and 30% of untreated tumors) with KU758 and KU711 treatment, respectively, we are able to demonstrate statistical significance only between KU758 and 17‐AAG as well as between all the three drugs (KU711, KU758, and 17‐AAG) and control untreated mice due to small sample size. Further steps in this investigation merit a large‐scale translational animal study with patient‐derived xenografts. Additionally, due to the ability of C‐terminal HSP90 inhibitors to specifically target TICs, it would be exciting to evaluate possible synergistic effects of these agents in combination with standard of care chemotherapy drugs for treatment of TNBC.

## 5 Conclusion

We conclude that C‐terminal HSP90 inhibitors are potent novel therapeutics against TNBC *in vitro* and *in vivo* as they target TICs and block migration/invasion, EMT transition, and cellular self‐renewal. These exciting findings suggest the need to further investigate KU711 and KU758 as possible agents for clinical trial.

## Conflict of interest

The authors declare no conflict of interest.

## Author contributions

CS, PTG, BSJB, and MSC conceived the idea and designed the project. CS and MSC analyzed and interpreted the data. AZ and BSJB prepared the C‐terminal HSP90 inhibitors. CS, PTG, JB, AK, and DK performed the experiments and collected the data. GW and PTW helped with the histology. CS, TW, and MSC wrote the manuscript.
